# *In vivo* and *in vitro* effects of hyperplasia suppressor gene on the proliferation and apoptosis of lung adenocarcinoma A549 cells

This article has been retracted.

**DOI:** 10.1042/BSR20180391

**Published:** 2018-10-02

**Authors:** Zhen-Qing Sun, Gang Chen, Qiang Guo, He-Fei Li, Zhou Wang

**Affiliations:** 1 Department of Thoracic Surgery, Shandong Provincial Hospital Affiliated to Shandong University, Jinan 250021, P.R. China; 2 Department of Thoracic Surgery, Affiliated Hospital of Hebei University, Baoding 071000, P.R. China

**Keywords:** A549 cells, Apoptosis, Gene silencing, Hyperplasia suppressor gene, Lung adenocarcinoma, Proliferation

## Abstract

Lung adenocarcinoma is the most common subtype of non-small cell lung cancer (NSCLC). Hyperplasia suppressor gene (HSG) has been reported to inhibit cell proliferation, migration, and remodeling in cardiovascular diseases. However, there lacks systematic researches on the effect of HSG on the apoptosis and proliferation of lung adenocarcinoma A549 cells and data of *in vivo* experiments. The present study aims to investigate the effects of HSG gene silencing on proliferation and apoptosis of lung adenocarcinoma A549 cells. The human lung adenocarcinoma A549 cell was selected to construct adenovirus vector. Reverse transcription-quantitative PCR (RT-qPCR) and Western blot analysis were conducted to detect expressions of HSG and apoptosis related-proteins. Cell Counting Kit (CCK)-8 assay was performed to assess A549 cell proliferation and flow cytometry to analyze cell cycle and apoptosis rate. The BALB/C nude mice were collected to establish xenograft model. Silenced HSG showed decreased mRNA and protein expressions of HSG, and elevated A549 cell survival rates at the time point of 24, 48, and 72 h. The ratio of cells at G_0_/G_1_ phase and apoptosis rate decreased and the ratio of cells at S- and G_2_/M phases increased following the silencing of HSG. There were decreases of B cell lymphoma-2 (Bcl-2)-associated X protein (Bax), Caspase-3, and Caspase-8 expressions but increases in Bcl-2 induced by silenced HSG. As for the xenograft in nude mice, tumor volume increased, and apoptosis index (AI) decreased after HSG silencing. These results indicate that HSG gene silencing may promote the proliferation of A549 cells and inhibit the apoptosis. HSG may be a promising target for the treatment of lung adenocarcinoma.

## Introduction

Lung cancer is the leading cause of cancer-related deaths worldwide. It has approximately caused 158000 deaths in the United States in the year 2015 [1]. Lung adenocarcinoma is the most common histological type of lung cancer, accounting for 50% of the incidences of non-small cell lung cancer (NSCLC) [2], and usually occurs in the glandular epithelium of the lung periphery from either type II pneumocytes or bronchioalveolar stem cells [3]. Lung adenocarcinoma is frequently diagnosed at advanced stages, contributing to a no more than 16% overall 5-year survival rate [4]. Lung adenocarcinoma is characterized by the formation of a gland or a duct and a massive bronchial mucosa. It generally originates in the peripheral lung tissue [5]. The major risk factors for lung adenocarcinoma are smoking or passive smoking (passive smokers are at a higher risk comparatively), exposure to cigarette smoke, asbestos, chromium, or arsenic compounds [6]. People suffering from lung adenocarcinoma usually have a poor prognosis or can also develop a resistant disease easily. Hence, there is an urgent need for advanced and valid therapeutic options [7]. The current therapeutic approaches for lung cancers include surgical removal of the tumor and adjacent lymph nodes, radio, and chemotherapy, but with limited efficacy [8,9]. The mutations in genes are related to growth, invasion, and metastasis, which form the molecular genetic basis of malignant transformation and tumor progression [10]. Therefore, identifying key genes or targets related to tumorigenesis can lead us to a new phase of lung adenocarcinoma treatment.

Hyperplasia suppressor gene (HSG), also known as Mitofusin 2 (mfn2), localizes to the mitochondrial outer membrane, which contains one GTPase domain in its NH_2_-terminal region, one coiled-coil domain, two transmembrane spans, and one coiled-coil domain in the carboxy-terminal region [11,12]. HSG also plays a key role in mitochondrial fusion, trafficking, and mitophagy, thus regulating mitochondrial morphology and function [13]. Moreover, HSG is a strong suppressor of cell proliferation both *in vitro* and *in vivo*, which is mediated by the suppression of mitogen-activated protein kinase signaling and cell-cycle arrest [14]. In addition, the pro-apoptotic function of HSG in various malignancies, such as hepatocellular and gastric cancers, was also taken into consideration and researched on [15,16]. Another study focussing on the effects of HSG on the lung cancer cell line A549 and colon cancer cell line HT-29 has found that adenovirus-expressing human HSG induces apoptosis in cancer cells [17]. Despite strong correlative evidence that HSG suppresses tumorigenesis, this has yet to be rigorously demonstrated *in vivo*. Therefore, the goal of the present study is to experiment and investigate the effect of HSG gene silencing on apoptosis and proliferation of lung adenocarcinoma A549 cells *in vitro* and *in vivo*, which is achieved by constructing the adenovirus vector and xenograft in nude mice.

## Materials and methods

### Cell culture

The human lung adenocarcinoma A549 cells, acquired from Chinese Academy of Sciences, Shanghai Institute Cell Bank, were stored in a RPMI 1640 culture medium (Gibco Company, Grand Island, NY, U.S.A.), containing 10% FBS for incubation at 37°C in a 5% CO_2_ incubator. Once the cells reached a confluence of approximately 80%, they were passaged. Following the removal of waste liquid, cells were washed twice by phosphate-buffered solution (PBS) and treated with 0.25% trypsin. Next, cells were made into suspension in RPMI 1640 culture medium containing 10% FBS. Then, cells were seeded into new culture bottles or plates at a certain density, and the cells that were at logarithmic phase were obtained for usage in further experimental analysis.

### Construction of lentiviral vector carrying *HSG* gene

HSG-specific interference RNAi sequence and the sequence of negative control (NC) were designed and synthesized by Shanghai Genechem Co., Ltd. (Shanghai, China): 5′-CAAAGGTTACCTATCCAAA-3′; 5′-TTCTCCGAACGTGTCACGT-3′. The lentiviral vector combined with packaging plasmid vector was co-transfected into 293T cells (Chinese Academy of Sciences, Shanghai Institute Cell Bank, Shanghai, China) by using Lipofectamine 3000 (Invitrogen Inc., Carlsbad, CA, U.S.A.). After culturing for 48 h, the supernatant was finally collected. High concentration virus cluster was obtained using the centrifugal ultrafiltration device and then titer determination was conducted. The infection was conducted when the multiplicity of infection (MOI) reached 20. A549 cells were firstly added into polybrene (Invitrogen Inc., Carlsbad, CA, U.S.A.). The cells at logarithmic phase were made into cell suspension and inoculated in a 24-well plate. When cell confluence reached approximately 15%, taking MOI value as reference, cells were added with an appropriate amount of virus and kept under observation after 12-h cultivation. If there was no definite cytotoxicity found, the medium was replaced after another cultivation for 12 h; otherwise, replaced immediately. After 3 days of infection, the infection efficiency were calculated with a fluorescence microscope. The vector with over 80% infection efficiency was selected for further experiments.

### Cell grouping and observation

Cells were assigned into the blank, siRNA against NC (si-NC), and siRNA against HSG (si-HSG). After detachment, cells at logarithmic phase were inoculated into six-well plates. Once the cells adhered to the wall, they were grouped as mentioned above. And then, cells were cultured in an incubator at 37°C with 5% CO_2_. After 4 h, the culture medium was changed, and the next experiment was performed after culturing for 24–72 h. After 48 h of culturing, cells were observed under an inverted microscope.

### Reverse transcription-quantitative PCR

The total RNA of cells in each group was extracted according to the instructions on kit (Qiagen, Valencia, CA, U.S.A.). The UV spectrophotometer was used to detect the optical density (OD) value (260/280) of extracted RNA and the concentration of RNA was calculated. Samples were stored at −80°C for preparations. The reverse transcription of cDNA was conducted in accordance with the instructions on kit (Qiagen, Valencia, CA, U.S.A.). Based on the gene published by Genbank database, Primer 5.0 primer design software was adopted and the sequences are shown in Table 1. All of the primers were synthesized by Shanghai Sangon Biological Engineering Technology & Services Co., Ltd. (Shanghai, China). Reverse transcription-quantitative PCR (RT-qPCR) reaction systems were 20 μl, including 10 μl SYBR Premix ExTaq, 0.4 μl Forward Primer, 0.4 μl Reverse Primer, 0.4 μl ROX Reference Dye II, 2 μl DNA template, and 6.8 μl ddH_2_O. Reaction conditions were as follows: pre-degeneration at 95°C for 30 s, 45 cycles of degeneration at 95°C for 20 s, and annealing/extension at 60°C for 20 s. Glyceraldehyde-3-phosphate dehydrogenase (GAPDH) was regarded as the internal reference and solubility curve was utilized to assess the reliability of PCR results. The collected *C*_T_ value (the threshold of the amplification curve) helped to calculate the relative expression of target gene according to 2^−ΔΔ*C*^_t_ [17].

**Table 1:** Primers used in RT-qPCR

Gene	Upstream (5′–3′)	Downstream (5′–3′)
*HSG*	CTCTCGATGCAACTCTATCGTC	TCCTGTACGTGTCTTCAAGGAA
*Caspase 3*	CATGGAAGCGAATCAATGGACT	CTGTACCAGACCGAGATGTCA
*Caspase 8*	TTTCTGCCTACAGGGTCATGC	GCTGCTTCTCTCTTTGCTGAA
*Bax*	CCCGAGAGGTCTTTTTCCGAG	CCAGCCCATGATGGTTCTGAT
*Bcl-2*	TGTTAGTGGAGAACATAAGTGGC	TGAATGGTGCTTGGTACAATCAT
*GADPH*	GGAGCGAGATCCCTCCAAAAT	GGCTGTTGTCATACTTCTCATGG

Abbreviations: Bax, Bcl-2-associated X protein; Bcl-2, B cell lymphoma-2.

### Western blot analysis

Protein of each group was extracted and its concentration was detected according to the instructions of BCA kit (Wuhan Boster Biological Technology Co., Ltd., Wuhan, Hubei, China). The extracted protein was added to the loading buffer and boiled at 95°C for 10 min, after which each well was added with 30 μg loading buffer. Protein separation was conducted with 10% polyacrylamide gel (Wuhan Boster Biological Technology Co., Ltd., Wuhan, China) on the electrophoretic voltage which was changed from 80 to 120 V. The wet transmembrane was performed at 100 mV for 45–70 min, and then the proteins were transferred on to the PVDF membrane. Subsequently, the samples were blocked by 5% BSA at room temperature for 1 h. Primary antibody HSG (1:1000), Caspase-3 (1:1000), Caspase-8 (1:1000), Bcl-2-associated X protein (Bax) (1:1000), B cell lymphoma-2 (Bcl-2) (1:1000; Abcam Inc., Cambridge, MA, U.S.A.), and GAPDH (1:1000; Santa Cruz Biotechnology, Inc., Santa Cruz, CA, U.S.A.) were added at 4°C for one night. The next day, protein samples were washed with Tris(-HCl)-buffered saline + Polysorbate 20 (Tween 20) (TBST) three times (5 min/time) and secondary antibody was added for 1-h incubation at room temperature, after which, the membrane was washed thrice (5 min/time) and chemiluminescence reagent was used for developing. GAPDH was used as the internal reference. The Bio-Rad Gel Dol EZ imager (Bio-Rad, Inc., Hercules, CA, U.S.A.) was applied for developing. ImageJ software was used to conduct Grey value analysis of target band.

### Cell counting kit-8 assay

The cell counting kit (CCK-8) (Dojindo Laboratories, Kumamoto, Japan) was selected for the assessment of A549 cell survival. After detachment using 0.25% trypsin, cells (10^5^ cells/ml) at logarithmic phase were seeded into a 96-well plates with 10^4^ cells/well (100 μl). After the treatment, the marginal wells were filled with PBS and then the samples collected were stored in an incubator for cell adherent. Once cell confluence reached up to 80%, the cells were treated according to the above grouping ways with six parallel wells set in each group. At the time point of 24, 48, and 72 h, each well was incubated with 10 μl CCK-8 solution in a 4°C refrigerator for 1–4 h. A microplate reader (Thermo Fisher Scientific, California, U.S.A.) was employed to measure the OD value at 450 nm. The above processes were repeated for three times and the mean OD value was obtained. Cells survival rate = OD _the experimental group_/OD _the blank group_.

### Flow cytometry of propidium iodide staining

First, A549 cells were fixed in ice absolute ethyl alcohol at 4°C for one night. Having been washed with PBS, cells were then centrifuged at 447.2×***g***. The supernatant was discarded. Each sample was added with 500 μl 1× FACS buffer (PBS, 0.1% BSA, and 0.01% NaN_3_) and 2.5 ml Rnase A (10 mg/ml) for complete mixture, followed by standing at room temperature for 15 min. Then, 25 μl propidium iodide (PI) (1 mg/ml; Beyotime Biotechnology Co., Shanghai, China) was added into each sample for 15-min incubation devoid of light at room temperature. Cell cycle was detected with a FACSCanto II flow cytometer (Becton, Dickinson and Company, NJ, U.S.A.).

### Flow cytometry of annexin V-FITC double staining

Annexin V kit was utilized for the detection of A549 cell apoptosis. The cultured cell solution in the six-well plates was extracted into centrifugation tubes and it was washed by PBS, and then 0.25% trypsin was used to treat the cells. After the cells were triturated, the digested solution was collected and the cells were added into the above culture solution for centrifugation at 12000 rpm at 4°C for 5 min. Then the supernatant was abandoned and the remaining cellular precipitation was collected. Samples were made into resuspension solution (50–100 thousand) by PBS, after which centrifugation was conducted for 5 min and the supernatant was removed. Then Annexin V-FITC (195 μl) was added for resuspension. Later, 5 μl of Annexin V-FITC was added and mixed for incubation of cells (in the dark) at room temperature for 10 min. After 5 min of centrifugation, the supernatant was discarded, after which, 190 μl Annexin V-FITC binding buffer and 10 μl PI staining solution were added. Ice-bath was conducted after the complete mixture. The flow cytometer (Becton, Dickinson and Company, NJ, U.S.A.) was utilized to detect the A549 cell apoptosis. The early apoptosis, late apoptosis, and survival cells were shown in the right lower quadrant, right upper quadrant, and left lower quadrant, respectively. Apoptosis rate = early apoptosis rate + late apoptosis rate.

### Construction of *in vivo* animal model

The animal experiments were approved by the ethics committee of Shandong Provincial Hospital Affiliated to Shandong University. A total of 18 female BALB/C nude mice, weighing 180–200 g and ageing 3–5 months old, were purchased from Shanghai Laboratory Animal Center (SLAC) Co., Ltd. (Shanghai, China). All mice were kept in a specific pathogen free (SPF) animal laboratory with maintained humidity and temperature. After 14-day adaptive feeding, the tumor formation assay in nude mice was performed. The A549 cells, stably transfected with adenovirus vector, were randomly assigned into the blank group, the si-NC group, and the si-HSG group (with six mice in each group). Cells at logarithmic phase were obtained and the cells concentration was adjusted to 5 × 10^7^ cells/ml on counting plates. The right underarm skin of nude mice was sterilized by alcohol on superclean benches. According to the ways of grouping, subcutaneous injection of 100 μl (5 × 10^6^) cells was conducted. There was an obvious piciu at the injection site. The growth of tumor was observed everyday after inoculation. On the seventh day after inoculation, callosity of rice-size was noted at the subcutaneous injection site, indicating that the inoculation was successful. The maximum diameter and vertical width of subcutaneous tubercle in nude mice were measured every 5 days after inoculation. The tumor volume was calculated and the growth curve was drawn accordingly. Tumor volume (cm^3^) = ab^2^/2 (a: maximum diameter; b: minimum diameter). On the 32nd day after inoculation, the nude mice were killed and the tumor was separated and weighted for further experiment.

### Immunohistochemistry

Tumor tissues were fixed in formalin and conventionally embedded in paraffin. Samples were made into 3-μm sections and xylene–alcohol gradient dehydration was conducted. Antigen retrieval was done by citrate solution (pH = 7.2–7.4), after which primary antibody HSG (1:500) was added at 4°C overnight. After 1-h incubation at 37°C, all the samples were washed by PBS (0.01 mol/l) and biotin-labeled secondary antibody working solution (Wuhan Boster Biological Technology Co., Ltd., Wuhan, China) was added for incubation at 37°C for 30 min. After developing for 10-min, using diaminobenzidine (DAB), the samples were counterstained with Hematoxylin, dehydrated with alcohol gradient, sealed in neutral balsam, and observed under a light microscope. The HSG-positive reactant was presented as brown granules in cell cytoplasm and nucleus. Immunohistochemistry sections were collected and observed under a microscope (400×). The average OD value was calculated by ImagePro Plus software, after which the statistical analysis was conducted [18].

### TdT-mediated dUTP nick-end labeling staining

The TdT-mediated dUTP nick-end labeling (TUNEL) kit (Beyotime Biotechnology Co., Beijing, China) was applied to detect the tumor tissues and calculate the apoptosis index (AI). Appropriate concentration and amount of protease K was added on to the paraffin sections for 30-min incubation at 37°C, after which, the samples were washed with PBS for five times. The section samples were shaken in 0.1% Triton X-100 buffer for 15 min, and then they were washed another five times with PBS containing 0.05% Tween 20 (PBST). According to the instructions on the kit provided, TUNEL solution was prepared and added on to the tumor tissues. After 60-min water bath at 37°C, samples were washed with PBST for five times. Following the addition of relevant antibodies, incubation of samples was performed devoid of light at 37°C for 30 min. Then, peroxidase (POD) was used for signal transduction. Developed by DAB, samples were washed with running water, cleared by xylene, and hydrated by gradient alcohol hydration (100 to 60%) (each process was conducted for 5 min). After that, samples were fixed in neutral resins and air dried for 12 h, followed by observation under a light microscope. Five visions of each section were selected under a light microscope (400×), based on which, the number of positive cells and total cells was calculated. AI = positive cells number/total cells number.

### Statistical analysis

Data were analyzed using the statistical package for the social sciences (SPSS) version 21.0 (IBM Corp. Armonk, NY, U.S.A.). Measurement data were displayed as mean ± S.D. Kolmogorov–Smirnov method was used to test the normality of data. One-way ANOVA with Tukey post hoc test was used for comparisons amongst groups. Dunns’s multiple comparison post hoc in Kruskal–Wallis test was performed for data that did not pass the normality test. Cell proliferation and cell cycle data were measured by repeated ANOVA. *P*<0.05 was regarded as statistically significant and different.

## Results

### HSG silencing reduces mRNA and protein expression of HSG and shows good morphology of lung adenocarcinoma A549 cells *in vitro*

After the construction of lentivirus vector for si-HSG, the mRNA and protein expression of HSG in each group were detected by RT-qPCR and Western blot analysis. Compared with the blank group, no significant difference of *HSG* mRNA expression was observed in the si-NC group (*P*>0.05), but *HSG* mRNA expression in the si-HSG group decreased by 38% (*P*<0.05) (Figure 1A). Western blot analysis further indicated that HSG protein expression was significantly down-regulated by 46% in the si-HSG group as compared with that in the blank group (*P*<0.05). No significant difference in the mRNA and protein expression of HSG was noted between the si-NC group and the blank group (*P*>0.05) (Figure 1B,C). Based on these results, it could be concluded that mRNA and protein expressions of HSG were decreased in the si-HSG group. The morphology of A549 cells after a span of 48-h culturing was observed under an inverted microscope. For the blank and NC groups, cells were stumped to the wall in the shape of oval and fusiform, and they were then connected closely and grew well with optimum bright cytoplasm and fast expansion rate. In comparison with the blank and NC groups, within the si-HSG group, the volume of the cells was found to be smaller, cell gap to be wider, and some cells were swollen, broken, shedding, and necrotic (Figure 1D–F).

**Figure 1:** HSG silencing reduces mRNA and protein expression of HSG and shows good morphology of lung adenocarcinoma A549 cells *in vitro* (**A**) *HSG* mRNA expression in each group detected by RT-qPCR; (**B**) HSG protein expression in each group detected by Western blot analysis; (**C**) protein bands of HSG protein expression in each group after Western blot analysis. Both experiments were repeated three times, the measurement data were analyzed by one-way ANOVA; *n*=6 per group; *, compared with the blank group, *P*<0.05. (**D–F**) Morphology of A549 cells after 48-h culturing observed with an inverted microscope (×100).

### HSG silencing enhances lung adenocarcinoma A549 cell viability and cycle entry, but inhibits apoptosis *in vitro*

The effects of HSG silencing on A549 cells proliferation were detected by CCK-8 assay. Compared with the blank group, no significant difference was noted in the si-NC group in terms of the cell proliferation rates at 24, 48, and 72 h (all *P*>0.05). The si-HSG group showed significant increased cell survival rates at 24, 48, and 72 h in comparison with those in the blank group (all *P*<0.05). Comparison between different time points indicated that cell proliferation rates at the time points of 24, 48, and 72 h significantly decreased as compared with that in the 0 h (all *P*<0.05). Compared with the cell proliferation rate at 24 h, the time points of 48 and 72 h showed a significant increase in cell proliferation rates (both *P*<0.05). Comparison between the time points of 48 and 72 h revealed significantly higher cells proliferation rate at 72 h (*P*<0.05), shown in Figure 2A. In order to explore and study the effect of HSG on the cell cycle and apoptosis of lung adenocarcinoma A549 cells, flow cytometry of PI staining and Annexin V-FITC double staining was conducted. Based on the obtained results (Figure 2B–E), the si-HSG group showed significantly lower ratio of cells at G_0_/G_1_ phase and increased ratio of cells at G_2_/M and S phases than the blank group (*P*<0.05). There was no significant difference between the si-NC group and the blank group in terms of cell ratio at G_0_/G_1_, S, and G_2_/M phases (all *P*>0.05), indicating that down-regulation of HSG expression could arrest less cells at G_0_/G_1_ phase, enhance the ratio of cells at S and G_2_/M phases, and thus, promote the proliferation of A549 cells. The effects of HSG silencing on apoptosis of A549 cells were detected by flow cytometry. There were many early apoptoses and late apoptoses in the blank and si-NC groups. Significant decreases in early apoptosis and late apoptosis of A549 cells were observed in the si-HSG group. Compared with the blank group, the si-HSG group showed significant decrease in cell apoptosis rate (*P*<0.05). No significant difference between the blank group and the si-NC group was noted in terms of cell apoptosis rate (*P*>0.05) (Figure 2F–I). The abovementioned results demonstrate that poor expression of HSG enhances lung adenocarcinoma A549 cell proliferation and cycle entry, but inhibits apoptosis *in vitro*.

**Figure 2:** HSG gene silencing inhibits the proliferation, and promotes apoptosis of A549 cells (**A**) Cell proliferation of the A549 cell in each group assessed by CCK-8 assay; (a) within one group compared with 0 h, *P*<0.05; (b) within one group compared with 28 h, *P*<0.05; (c) within one group compared with 48 h, *P*<0.05. * among multiple groups compared the blank group, *P*<0.05. (**B–D**) Cell cycle distribution of the A549 cell in each group determined by flow cytometry; (**E**) cell cycle rate of the A549 cell in each group; (**F–H**) cell apoptosis of A549 cells in each group measured by flow cytometry; (**I**) statistical analysis of (F–H). All experiments were repeated three times, and the measurement data were analyzed by one-way ANOVA; *n*=6 per group; *, compared with the blank group, *P*<0.05.

### HSG silencing decreases Bax, Caspase-3, and Caspase-8 expressions and increases Bcl-2 expression

The effects of HSG silencing on the expressions of cell apoptosis-related proteins were detected by carrying out RT-qPCR and Western blot analysis. In comparison with the blank group, the si-NC group was noted showing no remarkable difference in terms of the mRNA and protein expressions of Bax, Caspase-3, Caspase-8, and Bcl-2 (all *P*>0.05). The si-HSG group showed significantly decreased mRNA and protein expressions of Bax, Caspase-3, and Caspase-8 but increased *Bcl-2* mRNA and protein expression in the si-HSG group as compared with the blank group (all *P*<0.05) (Figure 3). Based on the results, we came to the conclusion that poor expression of HSG decreased mRNA and protein expressions of Bax, Caspase-3, and Caspase-8, but increased *Bcl-2* mRNA and protein expression.

**Figure 3:** HSG silencing decreases Bax, Caspase-3, and Caspase-8 expressions and increases Bcl-2 expression (**A**) mRNA expressions of Bax, Caspase-3, Caspase-8, and Bal-2 by RT-qPCR; (**B**) protein expressions of Bax, Caspase-3, Caspase-8, and Bal-2 by Western blot analysis; (**C**) protein bands of Bax, Caspase-3, Caspase-8, and Bal-2 after Western blot analysis. Both experiments were repeated three times, and the measurement data were analyzed by one-way ANOVA; *n*=6 per group; *, compared with the blank group, *P*<0.05.

### Repression of HSG increases the tumor growth and weight of lung adenocarcinoma A549 cells and inhibits tumor apoptosis *in vivo*

After the xenografts in nude mice succeeded, the tumor volume was measured every 5 days and tumor growth curve was drawn. According to the results, compared with the blank group, no significant difference in tumor volume and weight at each time point were seen in the si-NC group (all *P*>0.05), while the si-HSG group showed significant increase in tumor volume and weight at each time point (all *P*<0.05). The tumor volume and weight of each group significantly decreased over time (Figure 4A–C). It is suggested that the silencing of HSG increased the tumor growth and weight of lung adenocarcinoma A549 cells. The protein expression of HSG in tumor tissues of each group was detected by immunohistochemistry. The positive reactant of HSG presented as brown granules in cell plasma and cell nucleus. Based on the mean OD value of each group, no significant difference of HSG protein expression was noted between the blank and si-NC groups (*P*>0.05). In comparison with the blank group, HSG protein was significantly decreased in the si-HSG group (*P*<0.05) (Figure 4D–G). The results revealed that HSG protein was significantly decreased in tumor tissues in the si-HSG group. In order to further investigate the role of HSG in apoptosis *in vivo*, TUNEL staining was performed. According to the TUNEL staining results, the apoptotic cells mainly presented as clay-bank dense granules in cell nucleus. Few apoptotic cells were observed in the blank and si-NC groups. The si-HSG group showed much fewer apoptotic cells. The statistical analysis indicated that no significant difference of AI was noted between the blank and si-NC groups (*P*>0.05). When compared with the blank group, the si-HSG group revealed significantly decreased AI (*P*<0.05) (Figure 4H–K). Based on these findings, it could be concluded that the silencing of HSG represses tumor apoptosis of lung adenocarcinoma A549 cells *in vivo*.

**Figure 4:** Repression of HSG increases the tumor growth and weight of lung adenocarcinoma A549 cells and inhibits tumor apoptosis *in vivo* (**A**) Tumor growth of nude mice in each group; (**B**) tumor weight of nude mice in each group; (**C**) statistical analysis of tumor weight of nude mice at the 32nd day; (**D**–**F**) HSG expression in tumor tissue of each group by immunohistochemistry (×200); (**G**) OD value of HSG protein in each group; (**H**–**J**) A549 cell apoptosis in tumor tissue of each group by TUNEL staining (×400); (**K**) the histogram showing cell apoptosis rate in each group. All experiment were repeated three times, and the measurement data were analyzed by one-way ANOVA; *n*=6 per group; *, compared with the blank group, *P*<0.05.

## Discussion

Lung adenocarcinoma holds a high metastasis rate even at an early stage [5]. To the best of our knowledge, tumor metastasis is the leading death-cause amongst liver cancer patients [19]. A previous study indicates that the aberrant alternation of silenced tumor suppressor gene by promoter methylation is actually of great importance in the progression of small cell lung cancer (SCLC) [20]. RNAi-mediated gene silencing has already been evaluated as a potential therapy for a number of diseases in clinical trials [21]. Another study has reported that RNAi targetting STMN1 inhibits tumor growth *in vivo* in human gastric cancer cells [22]. The lentiviral vector is an ideal tool to transduce exogenous siRNA by suppressing the target gene both *in vivo* and *in vitro* [23]. Hence, the lentiviral vector for siRNA expression was a better-chosen option for the present study. the present study was performed in order to examine the effect of HSG gene silencing on apoptosis and proliferation of lung adenocarcinoma A549 cells. Based on the results, it has been proven that the HSG gene silencing is capable of promoting the proliferation rate and also inhibiting the cell apoptosis of human lung adenocarcinoma tumor A549 cells, which surely provides a new target for the treatment of lung adenocarcinoma.

Previous finding has suggested that adenovirus expression vectors may be able to allow higher HSG gene levels than plasmid expression vectors [17]. Wang et al. [24] also show that adenovirus-mediated HSG gene silencing promotes hepatocellular carcinoma cell viability and tumor growth in nude mice. According to the current study, it has been suggested that the silencing of HSG exhibits decreased *HSG* mRNA and protein expressions, along with decreased AI, increased tumor growth, and proliferation of A549 cells and also suppressed apoptosis of A549 cells. HSG is abundantly expressed in many organs and tissues, including brain, heart, liver, lung, skeletal muscle, and kidney, and can regulate cell proliferation, apoptosis, and differentiation of multiple cancer cell lines [25]. Hu et al. [26] have demonstrated that the expression of HSG inhibits hepatocellular carcinoma cell proliferation and also induces apoptosis via Bax, and adenovirus-mediated HSG down-regulation markedly builds up the growth of subcutaneous tumors in nude mice both *in vivo* and *in vitro*. Furthermore, HSG/Mfn2, a newly found gene correlated with hypertension, was once reported to be dramatically down-regulated in hyper-proliferative vascular smooth muscle cells [27]. HSG also shows inhibitory roles in the cell proliferation of colorectal and breast cancers [28,29]. A549 cells with HSG silencing via Crispr/Cas9 fundamentally promotes colony formation, cell proliferation, and invasion of cancer cells both *in vitro* and *in vivo* [30]. Another study indicates that HSG expression is reduced in human lung adenocarcinoma tissues, while HSG deficiency in A549 cells increases cell proliferation, inhibits cell apoptosis, and enhances tumor growth [31]. Therefore, HSG may be a contributor to the development of lung adenocarcinoma.

Additionally, the present study quite clearly revealed that silenced HSG down-regulated the expression of Bax, caspase-3, and caspase-8 and up-regulated Bcl-2. The Bcl-2 gene family, including Bcl-2 and Bax, plays key roles in apoptosis regulation, where Bcl-2 promotes anti-apoptotic and Bax has an apoptosis function [32]. Besides, Bax is a pro-apoptosis protein and it co-localizes with HSG during apoptosis [17]. Tubeimoside-1 functions as an apoptotic promoter in A549 cells by declining the expression of Bcl-2 and inclining the expression of Bax [33]. Caspase family proteins are prominent regulators during different phases of the apoptotic pathway [34]. Guo et al. [35] have confirmed that HSG plays a key role in mitochondrial fusion, which is principally mediated by inhibition of Akt signaling, and can increase mitochondrial Bax/Bcl-2 ratio, cytochrome c release, and activated caspases-9 and caspase-3; and HSG-induced apoptosis can be blocked by the overexpression of an active phosphoinositide 3-kinase mutant or activation of caspases-8. Chen et al. [36] have reported that overexpressed XAF1 suppresses cell proliferation and also promotes cell apoptosis in human lung adenocarcinoma cell line A549, thereby activating the cleavage of apoptosis-associated proteins Caspase-3 and Caspase-8. As a tumor suppressor, the mutations of p53 are the most prevalent molecular genetic abnormalities in lung cancer [37]. It maintains genomic stability and controls cell apoptosis [38]. HSG, also known as Mfn2, is reported to be a target gene of p53, and *Mfn2* mRNA and protein levels are up-regulated in a p53-dependent manner [39].

## Conclusion

To sum up, the present study establishes the adenovirus vector for HSG and nude mice xenograft model, and finds that HSG gene silencing can enhance proliferation and suppress apoptosis of lung adenocarcinoma A549 cells. HSG may be a promising target for the treatment of lung adenocarcinoma. Yet, after surveying quite a bit of additional studies it can also be believed that with various lung adenocarcinoma cell lines and large-scale experiments, it is imperative to regulate the specific role of HSG in lung adenocarcinoma. Ultimately, further studies on the functions of HSG, in detail, would be certainly beneficial for oncotherapy and in the process of doing so.

## Abbreviations

AI: apoptosis index
Bax: Bcl-2-associated X protein
Bcl-2: B cell lymphoma-2
CCK-8: cell counting kit
DAB: diaminobenzidine
GAPDH: glyceraldehyde-3-phosphate dehydrogenase
HSG: hyperplasia suppressor gene
JNK: c-jun NH2-terminal kinase
mfn2: mitofusin 2
MOI: multiplicity of infection
NC: negative control
NSCLC: non-small cell lung cancer
OD: optical density
PBS: phosphate-buffered solution
PBST: PBS containing 0.05% Tween 20
PI: propidium iodide
RT-qPCR: reverse transcription-quantitative PCR
si-NC: siRNA against NC
STMN1: stathmin
TUNEL: TdT-mediated dUTP nick-end labeling
